The article "Synthesis of efficient cobalt–metal organic framework as reusable nanocatalyst in the synthesis of new 1,4-dihydropyridine derivatives with antioxidant activity" was retracted in 2023. Reasons: signs of a paper mill; concerns about the authorship.

# Synthesis of efficient cobalt–metal organic framework as reusable nanocatalyst in the synthesis of new 1,4-dihydropyridine derivatives with antioxidant activity

**DOI:** 10.3389/fchem.2022.932902

**Published:** 2022-09-08

**Authors:** Omar dheyauldeen Salahdin, Indrajit Patra, Mohammad Javed Ansari, Samar Emad Izzat, Khusniddin Fakhriddinovich Uktamov, Mohammed Kadhem Abid, Ahmed B. Mahdi, Ali Thaeer Hammid, Yasser Fakri Mustafa, Himanshu Sharma

**Affiliations:** ^1^ Al-maarif University College, Medical Laboratory Techniques Department, Anbar-Ramadi, Iraq; ^2^ An Independent Researcher, PhD from NIT Durgapur, Durgapur, West Bengal, India; ^3^ Department of Pharmaceutics, College of Pharmacy, Prince Sattam Bin Abdulaziz University, Al-kharj, Saudi Arabia; ^4^ Al-Nisour University College, Baghdad, Iraq; ^5^ Senior teacher at “Economic security” Department, Tashkent State University of Economics, Tashkent, Uzbekistan; ^6^ Department of Anesthesia, College of Health and Medical Technology, Al-Ayen University, Thi-Qar, Iraq; ^7^ Anesthesia Techniques Department, Al-Mustaqbal University College, Babylon, Iraq; ^8^ Computer Engineering Techniques Department, Faculty of Information Technology, Imam Ja’afar Al-Sadiq University, Baghdad, Iraq; ^9^ Department of Pharmaceutical Chemistry, College of Pharmacy, University of Mosul, Mosul, Iraq; ^10^ Department of Computer Engineering and Applications, GLA University Mathura, Uttar Pradesh, India

**Keywords:** cobalt–metal organic framework, catalytic activity, dihydropyridine, antioxidant activity, DPPH method

## Abstract

Efficient cobalt–metal organic framework (Co-MOF) was prepared via a controllable microwave-assisted reverse micelle synthesis route. The products were characterized by SEM image, N_2_ adsorption/desorption isotherm, FTIR spectrum, and TG analysis. Results showed that the products have small particle size distribution, homogenous morphology, significant surface area, and high thermal stability. The physicochemical properties of the final products were remarkable compared with other MOF samples. The newly synthesized nanostructures were used as recyclable catalysts in the synthesis of 1,4-dihydropyridine derivatives. After the confirmation of related structures, the antioxidant activity of derivatives based on the DPPH method was evaluated and the relationship between structures and antioxidant activity was observed. In addition to recyclability, the catalytic activity of Co-MOF studied in this research has remarkable effects on the synthesis of 1,4 dihydropyridine derivatives.

## 1 Introduction

So far, several kinds of materials including oxide structures (Wu et al., 2013), composites (Güemes et al., 2020), carbon nanotubes (Mohanta et al., 2019), and metal organic frameworks (MOFs) (Al-Rowaili et al., 2018) have been considered because of their desirable physicochemical properties. Among these materials, MOF crystalline nanostructures have been remarked with high specific surface area, small size distribution, and significant porosity (Ding et al., 2019). These novel crystalline nanostructures have been emerging as very promising functional materials for gas storage, separation, catalysis, sensing, and medicine because of their stable features (Chen et al., 2020; Wu et al., 2020). These unique features make the MOFs very attractive in versatile applications with deep domains (Shu et al., 2020; Turki Jalil et al., 2021).

MOF crystalline nanostructures are synthesized using various methods, which can be referred to as sol-gel (Tarzanagh et al., 2019), hydrothermal (Zhao et al., 2008), and coprecipitation methods (Rani et al., 2020). The choice of an environmentally friendly, controllable, and facile route that affects the physicochemical properties of final products is of great importance. Microwave and reverse micelle are green, fast, and facile procedures that affect the production of samples with high performance (Shu et al., 2020; Mirhosseini et al., 2021). The results obtained from previous studies show that microwaves can also affect the specific surface of MOF nanostructures (Ma et al., 2021). Because the specific surface area is an effective factor that facilitates the applications of the products in a different area, the synthesis of the MOF nanostructures via microwave-assisted revere micelle can be a critical synthesis route. Nifedipine and felodipine (Figure 1) by cerebral and ischemic activity are effective drugs in the treatment of Alzheimer’s disease. Nifedipine and felodipine contain 1,4-dihydropyridine nuclei. 1,4-Dihydropyridines nucleus is known in calcium channel agonist–antagonist modulation activities and used in cardiovascular diseases (Bossert et al., 1981; Bandgar et al., 2008; Singh et al., 2018).

**FIGURE 1:** Structure of Alzheimer’s disease drugs contain 1,4-dihydropyridine.

Examination of previous reports shows that several biological properties such as anti-lung cancer activity (Sharma et al., 2021a), antimicrobial properties (Mahinpour et al., 2018), antitubercular activity (Wang et al., 2019), and antioxidant activity (Anaikutti and Makam, 2020) have been reported from 1,4-dihydropyridine.

The most important method for the synthesis of 1,4-dihydropyridine was the application of dimedone, acetoacetate, aldehyde derivatives, and ammonium acetate using various catalysts (Calvino-Casilda and Martín-Aranda, 2020; Ali El-Remaily et al., 2021; Maleki et al., 2021).

In this research, efficient Co-MOFs were synthesized and used as recyclable catalysts in the synthesis of new 1,4-dihydropyridine derivatives. The advantages of nanoparticles used in this reaction include high productivity and shorter derivatives synthesis time.

The novelty of this work was the synthesis and reported efficient nanocatalyst in the synthesis of 1,4-dihydropyridine derivatives and the development of new derivatives of 1,4-dihydropyridine.

## 2 Experimental section

### 2.1 Materials and analysis devices

Co (III) nitrate pentahydrate (98.99%) and 2, 6-pyridine dicarboxylic acid (99.98%) were purchased from Merck. A surfactant agent as sodium dodecyl sulfate (SDS) (99.99%) and an oil phase as n-hexane (99.99%) were purchased from Sigma. All compounds used in this study were used as received, without further purification.

In the DMSO-*d*6 solutions, ^1^H and ^13^C-NMR spectra were recorded using Bruker FT-NMR Ultra Shield-250 spectrometer (250 and 75 MHz, respectively). Using the Kruss-type KSP1N melting point meter, the melting points of derivatives were determined and uncorrected.

### 2.2 Synthesis of cobalt–metal organic framework nanostructures

For a typical synthesis of Co-MOF nanostructures via microwave-assisted reverse micelle, a solution of Co (III) nitrate pentahydrate (0.3 mmol) and 2, 6-pyridine dicarboxylic acid (0.9 mmol) in 20 ml of double-distilled water is prepared. The mixture was then added to a related solution containing 0.03 mmol of SDS and 55 ml of n-hexane. The mixture was then added to the microwave bath and undergoes optimal conditions of time duration of 20 min, temperature of 30°C, and microwave power of 120 W. After 50 min, the red crystals of Co-MOF nanostructure are formed, separated by the centrifuge, and washed with DMF.

### 2.3 General procedure for the synthesis of 1,4-dihydropyridine derivatives (5a–h)

A mixture of 1 mmol aromatic aldehydes, 1 mmol dimedone (0.141 g), 1 mmol acetoacetate (methyl acetoacetate or ethyl acetoacetate), 1.2 mmol ammonium acetate (0.091 g), and 3 mg Co-MOF in 2 ml EtOH was stirred at 60°C. The reaction was monitored via thin-layer chromatography. After the completion of the reaction, 10 ml acetone was added to the mixture and cat isolated via nanofiltration. The solvent was then removed in a vacuum. In the end, the precipitates were recrystallized in ethanol.

Methyl 4-(2,6-dimethoxyphenyl)-2,7,7-trimethyl-5-oxo-1,4,5,6,7,8-hexahydroquinoline-3-carboxylate (5b).

^1^H NMR (DMSO-d6) *δ* = 0.75 (s, 3H, CH_3_), 0.97 (s, 3H, CH_3_), 1.95–1.97 (m, 2H, CH_2_), 2.16 (s, 3H, CH_3_), 2.45–2.46 (m, 2H, CH_2_), 3.52 (s, 3H, OCH_3_), 3.68 (s, 6H, OCH_3_), 5.21 (s, 1H, CH), 6.42 (d, 8.2 Hz, 2H, H-Ar), 6.79 (8.2 Hz, 1H, H-Ar), 8.79 (s, 1H, NH), ^13^C NMR (DMSO-d6) *δ* = 17.8, 24.7, 25.3, 28.7, 31.6, 38.9, 52.6, 54.7, 55.4, 56.3, 100.9, 103.6, 107.5, 123.2, 126.5, 142.7, 143.9, 149.9, 150.3, 191.6. Elemental analysis: Calcd for C_22_H_27_NO_5_: C, 68.55; H, 7.06; N, 3.63; O, 20.75. Found: C, 68.59; H, 7.09; N, 3.61; O, 20.71.

Methyl 4-(5-bromo-2-hydroxyphenyl)-2,7,7-trimethyl-5-oxo-1,4,5,6,7,8-hexahydroquinoline-3-carboxylate (5c).

^1^H NMR (DMSO-d6) *δ* = 0.82 (s, 3H, CH_3_), 1.01 (s, 3H, CH_3_), 1.76–1.79 (m, 2H, CH_2_), 2.32 (s, 3H, CH_3_), 2.52–2.53 (m, 2H, CH_2_), 3.76 (s, 3H, OCH_3_), 5.13 (s, 1H, CH), 6.62–6.64 (d, 8.4 Hz, 1H, H-Ar), 6.78–6.80 (d, 8.2 Hz, 1H, H-Ar), 6.91 (s, 1H, H-Ar), 9.12 (s, 1H, NH), 9.57 (s, 1H, OH), ^13^C NMR (DMSO-d6) *δ* = 17.2, 23.8, 24.5, 28.8, 31.2, 38.9, 48.5, 50.3, 52.5, 55.7, 101.4, 103.7, 107.1, 120.9, 124.8, 125.8, 143.9, 147.6, 152.1, 189.7. Elemental analysis: Calcd for C_21_H_24_BrNO_4_: C, 58.07; H, 5.57; N, 3.22; O, 14.73. Found: C, 58.10; H, 5.58; N, 3.21; O, 14.70.

Methyl 4-(2,6-dichlorophenyl)-2,7,7-trimethyl-5-oxo-1,4,5,6,7,8-hexahydroquinoline-3-carboxylate (5d).

^1^H NMR (DMSO-d6) *δ* = 0.94 (s, 3H, CH_3_), 1.03 (s, 3H, CH_3_), 1.96 (s, 2H, CH_2_), 2.25 (s, 3H, CH_3_), 2.52–2.53 (m, 2H, CH_2_), 3.01 (s, 3H, OCH_3_), 5.67 (s, 1H, CH), 6.72–6.75 (m, 3H, H-Ar), 9.03 (s, 1H, NH), ^13^C NMR (DMSO-d6) *δ* = 19.1, 23.9, 24.7, 29.3, 32.3, 38.7, 48.9, 50.1, 52.3, 55.6, 102.4, 103.5, 106.9, 123.4, 124.6, 135.8, 139.9, 146.1, 155.4, 193.7. Elemental analysis: Calcd for C_20_H_21_Cl_2_NO_3_: C, 60.92; H, 5.37; N, 3.55; O, 12.17. Found: C, 60.90; H, 5.38; N, 3.52; O, 12.20.

### 2.4 *In vitro* antioxidant activity

Antioxidant activities of derivatives on DPPH according to previously reported methods were evaluated (Beyzaei et al., 2018; Moghaddam‐Manesh et al., 2019). In a methanolic solution of DPPH (4 ml, 0.004% w/v), 1 ml of derivatives (concentrations of 25, 50, 75, and 100 μg/ml) was added and stood for 30 min at room temperature in darkness, and then, the absorbance was read against blank at 517 nm.

According to Eq. 1, percent inhibition (I %) of derivatives on free radical DPPH was calculated.

% of scavenging (1) = (A control − A sample) (A control) × 100.

A control: all the reagents except the test compound; A sample: absorbance of the test compound; Equation 1 is Calculation of % of scavenging. In antioxidant activity, tests were conducted in triplicate and their average was reported.

## 3 Results and discussion

### 3.1 Synthesis and characterization of cobalt–metal organic framework nanostructures

Figure 2A shows the thermal behavior of Co-MOF nanostructures synthesized using the effective microwave-assisted reverse micelle route. Furthermore, the results from the thermal behavior of the Co-MOF sample are presented in Table 1. According to these tables, the thermal stability of the Co-MOF product is approximately 388°C. This degree of stability is higher than that of various groups of materials such as nonporous material, fibrous compound, and ceramic polymer (Andrievski, 2014). In addition, the thermal stability of Co-MOF nanostructures synthesized in this study is higher than the sample synthesized in the previous study (Meng et al., 2013), which is related to the effective synthesis route developed in the present study. Because thermal stability is one of the effective factors in designing MOF nanostructures for application in various fields (Ding et al., 2019), the synthesis of Co-MOF samples with high thermal stability causes the potential development of these efficient materials.

**FIGURE 2:** Thermal curve **(A)**, SEM image **(B)**, N_2_ adsorption/desorption behaviour **(C)** and XRD patterns of Co-MOF nanostructures synthesized by microwave assisted reverse micelle route **(D)**.

**TABLE 1:** Thermal results of the Co-MOF samples synthesized by microwave assisted reverse micelle route.

Steps. No	Temperature (°C)	Probable composition of grp. Lost
I	76	Vanishing the adsorbed solvent
II	109	Evaporation of the trapped solvent
III	390	Micelle disintegration
IV	445	Ligand (linker) decomposition
V	522	Final decomposition

Figure 2B exhibits an SEM image of Co-MOF nanostructures synthesized via microwave-assisted reverse micelle route. As shown in this figure, the final structure of the Co-MOF nanostructures sample does not exhibit any evidence of particle agglomeration. The synthesis of samples with high surface stability as well as homogeneous morphology can be attributed to the optimal effects of the microwave-assisted reverse micelle method. In addition, based on the SEM image, the particle size distribution of products is in the form of one-dimensional nanostructures (average particle size of 50 nm), which confirms the nanostructure nature of the Co-MOF nanostructures. As an important result, Co-MOF products with a uniform surface and a narrow size distribution provide have great potential for medical applications (Moghadasi et al., 2021; Ghaffar et al., 2022; Kartika et al., 2022).

The adsorption/desorption isotherms of Co-MOF nanostructures fabricated via the microwave-assisted reverse micelle method are shown in Figure 2C. Based on this isotherm, the adsorption/desorption behavioral feature of the sample is similar to the fourth type of classical isotherms, which provides a high specific surface area for final products (Mirhosseini et al., 2021; Hachem et al., 2022; Sadeghi et al., 2022). Because the specific surface area is an effective parameter that affects the applications of the sample, this isotherm confirms the desired textural properties for the Co-MOF nanostructures. More details for BET characterization indicate a specific surface area of approximately 1700 m^2^/g for the Co-MOF nanostructure sample, which provides an effective surface interaction of the nanostructure with a reagent. In addition, the surface area of Co-MOF synthesized in this study is significantly higher than those in previous samples. The XRD patterns of Co-MOF synthesized in this study via microwave-assisted reverse micelle route are shown in Figure 2C. Based on the data, the related peaks were confirmed by previous samples. In addition, the wildness of XRD patterns was decreased, which confirmed the nanoscale distributions of peaks.

Figure 3 exhibits the FTIR spectrum of Co-MOF nanostructures synthesized via microwave-assisted reverse micelle route. According to this spectrum, the peak at approximately 3,500 cm^−1^ indicates the coordinated water in the Co-MOF structure. In addition, the frequency at approximately 3,200 cm^−1^ confirmed the presence of the carboxyl group in the final structure. The peak at approximately 3,000 cm^−1^ shows the stretch bond of C-H in products. The frequency at approximately 1,500 cm^−1^ confirmed the presence of the COO group in the Co-MOF nanostructures (Bakhshi et al., 2022). In addition, the absorption band at 1,400 cm^−1^ shows the stretch bond of (C-C) in the MOF sample. The frequency at approximately 900–700 cm^−1^ may be attributed to the bond Co-O in the final MOF nanostructures (Al-Attri et al., 2022).

**FIGURE 3:** FTIR spectrum of Co-MOF nanostructures synthesized by microwave assisted reverse micelle route.

According to the FT-IR spectrum and related configuration of ligand, Figure 4 was proposed for Co-MOF nanostructures.

**FIGURE 4:** Suggested formula for Co-MOF nanostructures synthesized by microwave assisted reverse micelle route.

### 3.2 Synthesis of 1,4-dihydropyridine derivative

1,4-Dihydropyridine derivative was synthesized based on Scheme 1.

**SCHEME 1:** Synthesis 1,4-dihydropyridine derivative by Co-MOF nanostructures.

**SCHEME 2:** Proposed mechanism for the synthesis 1,4-dihydropyridine derivative by Co-MOF nanostructures.

The optimization of reaction conditions such as solvent, amount of catalyst, and reaction temperature for the synthesis of 5a was investigated, and the results are presented in Table 2.

**TABLE 2:** Optimization conditions (solvent, amount of catalyst and temperature) in synthesis of 5a..

No	Product	Solvent	Amount of catalyst (mg)	Temperature (^o^C)	Time (min)	Yield (%)
1	5a	H_2_O	1	50	60	36
2	5a	H_2_O:EtOH (1:1)	1	50	60	54
3	5a	EtOH	1	50	20	83
5	5a	MeOH	1	50	60	31
6	5a	CH_3_CN	1	50	60	N. R
7	5a	EtOH	2	50	20	88
8	5a	EtOH	3	50	15	92
9	5a	EtOH	4	50	15	91
10	5a	EtOH	5	50	15	90
11	5a	EtOH	3	r. T	60	42
12	5a	EtOH	3	40	30	71
**13**	**5a**	**EtOH**	**3**	**60**	8	**95**
14	5a	EtOH	3	reflux	10	92

Ethanol, 60°C and 3 mg of Co-MOF nanostructures were obtained as the optimal solvent, temperature and amount of catalyst, conditions for synthesis 5a. In optimizing the amount of the catalyst, the amounts of 1, 2, 3, 4, and 5 mg of the catalyst were examined and the results showed that the amounts of 3, 4 and 5 mg give the highest efficiency and their results were slightly different. Therefore, the amount of 3 mg of catalyst was chosen as the optimal amount of catalyst.

The optimal conditions for synthesis 5a included ethanol as solvent, temperature of 60°C, and catalyst amount of 3 mg. In optimizing the amount of the catalyst, the amounts of 1, 2, 3, 4, and 5 mg of the catalyst were examined, and the results showed that the amounts of 3, 4, and 5 mg give the highest efficiency, and their results were slightly different. Therefore, the amount of 3 mg of catalyst was chosen as the optimal amount of catalyst.

In the optimal conditions, eight derivatives of 1,4-dihydropyridine were synthesized (Table 3) and three derivatives were new compounds (5b, 5c, 5d).

**TABLE 3:** Synthesis of 1,4-dihydropyridine derivatives (5a–h).

Entry	Product	R_2_	Structure	Time (min)	Yield (%)	Mp (°C)	
						Found	Reported
1	5a	Me		8	95	257–259	256–258 Aghaei-Hashjin et al. (2021)
2	5b	Me		30	72	215–217	New
3	5c	Me		36	87	220–222	New
4	5d	Me		25	83	235–237	New
5	5e	Et		10	93	258–260	255–257 Zabihzadeh et al. (2020)
6	5f	Et		25	75	217–219	220–223 Yousuf et al., 2020
7	5g	Et		45	91	227–228	226–228 Jadhvar et al. (2017)
8	5h	Et		20	86	241–243	243–245 Sharma et al. (2021b)

The proposed mechanism for the synthesis of derivatives was given in Scheme 2.

Based on previous reports, cobalt compounds and nanostructures containing cobalt have a high ability in the synthesis of heterocyclic and organic compounds. Cobalt can act as a Lewis acid in organic reactions (Kazemi et al., 2018; Rostami and Shiri, 2019; Moeini et al., 2021; Paudel et al., 2021). In the proposed mechanism, the Co-MOF nanostructures react as a Lewis acid and activate the carbonyl groups in terms of electron lethality in knoevenagel reaction and Michael’s incremental reaction on a proposed mechanism (I, II, III product number).

First, the form of enol daimedon with aldehyde by knoevenagel reaction product (I) was obtained. By contrast, during to reaction of ethyl acetate with ammonia product number (II) were obtained. With Michael’s incremental reaction between I and II, intermediate (III) was obtained, which becomes V. Then, during an intramolecular nucleophilic reaction and the replacement of nitrogen with oxygen, which occurs in form IV, and the removal of water, immunic product V was obtained.

At last, by changing the form of imine to amine, the final product was obtained.

Based on the results of Figure 5, the Co-MOF nanostructures that are used as catalysts have high recycling properties and can be reused six times without significant reduction in efficiency.

**FIGURE 5:** Reusability of Co-MOF nanostructures in synthesis 1,4-dihydropyridine derivatives.

There have been many reports on the use of different catalysts in the synthesis of 1,4-dihydropyridine, and Table 4 lists some of their most recent studies compared with the nanoparticles used in this study.

**TABLE 4:** Comparison of different catalysts in the synthesis methyl 4-(4-methoxyphenyl)-2,7,7-trimethyl-5-oxo-1,4,5,6,7,8-hexahydroquinoline-3-carboxylate (5a).

Entry	Cat	Time (min)	Temperature (°C)	Yield (%)
1	Mo@GAA-Fe_3_O_4_MNPs (10 mg) Aghaei-Hashjin et al. (2021)	15	90	95
2	BiFeO_3_ (5 mg) Singh et al. (2018)	3	100	93
3	Ti@PMO‐IL (0.2 mol%) Elhamifar et al. (2018)	26	60	93
4	Nickel containing ionic liquid (0.5 mol%) Elhamifar et al. (2017)	15	70	95
5	Co. MOF (3 mg) (this word)	8	60	95

The results were evaluated with ascorbic acid based on our previous reports (Moghaddam-Manesh et al., 2019).

As can be seen from the results of Table 3, the Co-MOF nanostructures studied in this project, in addition to high recyclability, can synthesize derivatives at a lower temperature and time with higher efficiency. In addition, a smaller amount of catalyst was used in the synthesis.

### 3.4 Antioxidant evaluation

The results of antioxidant activity of derivatives against DPPH free radical are given in Table 5. The IC_50_ values for 5a–h derivatives were 12.68, 13.86, 13.43, 13.98, 12.75, 14.91, 14.46, and 14.03 μg/m, respectively.

**TABLE 5:** Antioxidant activities of 1,4-dihydropyridine derivatives (5a–h).

Derivatives	(%) Scavenging concentrations (μg/ml)				IC50 (μg/ml)
	5	10	15	20	
5a	45	49	55	64	12.68
5b	46	49	52	57	13.83
5c	43	47	56	59	13.43
5d	40	43	55	59	13.98
5e	42	48	55	59	12.75
5f	39	43	51	56	14.91
5g	39	42	53	58	14.46
5h	41	45	54	58	14.03
Ascorbic acid	87.5	92.25	97.08	98.98	3.94

Based on the results of antioxidant activity, it was found that the antioxidant activity of the derivatives was close to each other, and not much difference was observed between IC_50_. Therefore, antioxidant activity does not depend on aldehyde derivatives, and the following mechanism (Figure 6) was proposed for the radical stability of DPPH.

**FIGURE 6:** Proposed mechanism for radical stability of DPPH by 1,4-dihydropyridine derivatives.

## 4 Conclusion

In this study, efficient Co-MOF nanostructures were developed via an efficient microwave-assisted reverse micelle route. The final products showed high thermal stability, significant porosity, and homogenous morphology. According to the FTIR spectrum, the suggested structures for products were presented. Co-MOF nanostructures were used as catalysts in the synthesis of 1,4-dihydropyridine derivatives. The use of Co-MOF nanostructures increased the efficiency and reduced the synthesis time of derivatives. Catalyst recyclability was another advantage of using Co-MOF nanostructures, and new 1,4-dihydropyridine derivatives were synthesized and identified in this study. In the following, the antioxidant activity of the derivatives was investigated and a proposed mechanism for the radical stability of DPPH using derivatives was presented.

## Data Availability

The original contributions presented in the study are included in the article/Supplementary Material; further inquiries can be directed to the corresponding author.
